The article "Anaerobic Treatment of Palm Oil Mill Effluent in Pilot-Scale Anaerobic EGSB Reactor" was retracted in 2018. Reason: duplicate publication.

# Anaerobic Treatment of Palm Oil Mill Effluent in Pilot-Scale Anaerobic EGSB Reactor

**DOI:** 10.1155/2015/398028

**Published:** 2015-06-18

**Authors:** Jin Wang, Qaisar Mahmood, Jiang-Ping Qiu, Yin-Sheng Li, Yoon-Seong Chang, Xu-Dong Li

**Affiliations:** ^1^College of Agriculture and Biology, Shanghai Jiao Tong University, Shanghai 200240, China; ^2^Department of Environmental Sciences, COMSATS Institute of Information Technology, Abbottabad 22060, Pakistan; ^3^Ronser Bio-Tech Sdn Bhd, C708, Metropolitan Square, Bandar Damansara Perdana, 47820 Petaling Jaya, Malaysia

## Abstract

Large volumes of untreated palm oil mill effluent (POME) pose threat to aquatic environment due to the presence of very high organic content. The present investigation involved two pilot-scale anaerobic expanded granular sludge bed (EGSB) reactors, continuously operated for 1 year to treat POME. Setting HRT at 9.8 d, the anaerobic EGSB reactors reduced COD from 71179 mg/L to 12341 mg/L and recycled half of sludge by a dissolved air flotation (DAF). The average effluent COD was 3587 mg/L with the consistent COD removal efficiency of 94.89%. Adding cationic polymer (PAM) dose of 30 mg/L to DAF unit and recycling its half of sludge caused granulation of anaerobic sludge. Bacilli and small coccid bacteria were the dominant microbial species of the reactor. The reactor produced 27.65 m^3^ of biogas per m^3^ of POME which was utilized for electricity generation.

## 1. Introduction

Palm oil industry is one of the most important types of agriculture based commerce in Malaysia and Indonesia. Malaysia covered about 5 million hectares of the palm cultivated area with 426 operating mills in 2011 [1]. Large quantity of water is required during the extraction process; consequently, the palm oil production generates huge quantity of palm oil mill effluent (POME). It is estimated that about 0.75 m^3^ of POME is generated when 1 ton of fresh fruit bunch (FFB) is processed [2]. POME is a concentrated yellow liquid with a distinct offensive odor and is characterized by high chemical oxygen demand (COD) and biochemical oxygen demand (BOD) in the range of 44,300–102,696 mg/L and 25,000–65,714 mg/L, respectively. The other characteristics include its acidic nature (pH 3.4–5.2), high salt and suspended solids (18,000–46,011 mg/L), and high Oil and grease (4000–9341 mg/L) contents [1]. POME can cause considerable environmental problems if discharged without any effective treatment.

Anaerobic digestion is one of the most widely employed biotechnologies for POME because it not only digests the high organic contents of wastewater but also generates renewable energy in the form of biogas. Various types of reactor configurations like closed-tank anaerobic digester, open digester tank, or covered lagoon have been widely used for anaerobiosis. Conventional facultative lagoons and open digesting tanks are the most commonly employed designs to treat POME. Although these processes require relatively little capital investment and operational energy, they require longer retention times usually in range of 20~60 days and extensive land area [2–5]. Additionally, enormous quantities of undigested suspended solids (SS) would gradually settle down at the bottom and occupy bulk of the lagoon area. Furthermore, the collection and utilization of produced biogas in these conventional anaerobic digesters are difficult which may escape into the atmosphere contributing to global warming.

Continuous stirred-tank reactor (CSTR) [6], up-flow anaerobic sludge blanket (UASB) [7], and up-flow solids reactor (USR) [8] are well-established anaerobic processes for the treatment of concentrated wastewaters with high COD-like POME. Additionally, a few improved high rate bioreactors such as the modified anaerobic baffled bioreactor (MABR) [9], the up-flow anaerobic sludge fixed-film (UASFF) reactor [10], and the advanced anaerobic expanded granular sludge bed (EGSB) [11] have also been tested for the treatment of POME. The results obtained from abovementioned studies indicated that advanced anaerobic digesters displayed better performance in POME treatment compared to conventional practices. However, pilot-scale or even industrial-scale implementation of any of the improved systems is still awaited.

The stability test of newly devised system before its industrial application is highly desirable. Two industrial-scale pilot EGSB reactors to treat POME were constructed and the first year performance was presented by Loh et al. [2] based on 10 hr daily operation. The present study reports the POME treatment efficiency and stability in EGSB during second year.

## 2. Materials and Methods

### 2.1. Experimental Setup

A Pilot-scale POME treatment plant was installed at Kilang Kelapa Sawit (KKS) Labu, Sime Darby, KM 16, 71900 Labu, Negeri Sembilan of Malaysia [2]. No specific permissions were required for these locations/activities and the field studies did not involve endangered or protected species there. The schematic diagram and photographic presentation of the EGSB reactor were shown in Figure 1. The steel tank of EGSB had diameter and height of 6 m and 16 m, respectively. The tanks were designed to operate in series using a set of valves, 2 dosing tanks; dissolved air flotation (DAF) was used to collect SS from EGSB effluent and partly recycled the anaerobic sludge back to EGSB.

The EGSB reactor was comprised of three sections: three-phase separator at the top, reactor body in the middle, and liquid distributor at the bottom. Ten sampling pipes were located in the middle section (reactor body) arranged at the intervals of 1 or 2 m each. The total volume of the reactor was 423.9 m^3^. Walls were covered with cotton acting as heat preservation layer. The temperature of the reactor was kept around 35°C during the study, which was suitable for anaerobic sludge during operation. The influent was pumped into the bottom of the reactor by a pump and the treated effluent exited at the top of the reactor.

The pilot-scale EGSB reactor was seeded with inoculum from open anaerobic ponds of local POME treatment plant. During early stages of start-up, the reactors were seeded with 10 g SS L^−1^ (6.5 g VSS (volatile suspended solids) L^−1^); after the intermittent operation for one year, it was kept at 20–40 g SS L^−1^ (15–30 g VSS L^−1^).

The EGSB reactors were operated at the hydraulic retention time (HRT) of 10 days, which was adjusted from 8 days based on the performance during previous year [2]. Its superficial hydraulic velocity was about 0.13 m h^−1^, while superficial airflow velocity was about 1.76 m h^−1^.

### 2.2. Characteristics of the POME

The open lagoon system in KKS Labu, Sime Darby, consisted of a cooling pond, an acidification pond, 2 anaerobic ponds, 2 facultative ponds, and a final discharge pond. Considering the current processing capacity of the mill, the overall HRT of lagoon was set above 100 days. Loh et al. [2] had presented the operational performance for the first year of the pilot-scale EGSB reactors based on 10 hr daily operation. The reactors were operated for 24 hr daily. The inlet POME was pumped from equalization tank after the pretreatment to remove oil.

A detailed account of the characteristics of POME from various sources was presented in Table 1. The POME from the palm oil pilot plant in KKS Labu (source b) had an obvious higher COD and suspended solids (SS) concentrations compared to normal POME (source a).

### 2.3. Analytical Methods

The wastewater characteristics like pH, COD, suspended solids (SS), volatile suspended solids (VSS), volatile fatty acid (VFA), and total alkalinity were analyzed according to the Standard Methods for Examination of Water and Wastewater [12]. BOD was analyzed based on the methods developed by DOE [13]. The microbiological features of the anaerobic granular sludge were studied using a scanning electron microscope (SIRION 200, FEI, USA) at 5 kV.

## 3. Results and Discussion

POME contained high oil and grease (O&G) and SS fractions. O&G and SS are generally known as obstacles for biological digestion; thus removal of O&G is prerequisite to ensure effective anaerobic treatment of POME. The recovered oil can be sold out as by-product. Following the oil separator tank (adopted to collect oil sludge), an equalization tank (EQ tank) was used as a buffer to make the operation stable. To control the influent temperature in the optimum mesophilic range (35 ± 2°C), a cooling tower was employed. POME was pumped from EQ tank to the dosing tanks where pH and temperature could be adjusted. During the pilot-scale test, caustic was not required to adjust pH as it was adjusted only by recycling part of anaerobic effluent.

The EGSB reactors were operated at HRT of 10 d. The data presented in Figure 2 and Table 2 suggested that anaerobic EGSB accomplished overwhelming COD reduction in spite of daily fluctuations in the influent characteristics. On average, COD decreased from 71179 to 12341 mg/L. After SS removal by DAF, the average COD was 3587 mg/L with COD removal efficiency of 94.89%. As half of the sludge from DAF was recycled to EGSB, it implied that half sludge was biodegraded during the operation.

The performance parameters of anaerobic EGSB and biogas production were presented in Table 3. The produced biogas was about 27.65 m^3^ per m^3^ POME. It approximated about 28 times based on laboratory studies [14]. The biogas production in EGSB was 52.7 m^3^/h or 0.44 m^3^ biogas/kg COD, at the rate of 15–21 m^3^ biogas per m^3^ POME [2]. The biogas composition was rather stable with 65–70% CH_4_, 25–36% of CO_2_, and 800–1500 ppm of H_2_S. The methane yield (0.29 to 0.31 m^3^ biogas (STP)/kg COD) obtained in the current study showed that the COD conversion as methane accounted for 82.9–88.6% of theoretical value (0.35 m^3^ biogas (STP)/kg COD). The biogas production was comparable and even better than previous reports [4, 10, 15]. The biogas was employed in electricity production after desulfurization.

EGSB reactors are gaining popularity and gradually replacing up-flow anaerobic sludge blanket (UASB) applications because of their higher loading rates. The successful operation of UASB and EGSB requires the granulation of anaerobic sludge. Sludge granulation is considered to be the most critical parameter affecting operational success of UASB and EGSB reactors [16]. In the past, continuous efforts have been put forth to accelerate anaerobic sludge granulation including addition of inert materials [17], organic polymers [18, 19], hybrid polymer [20], and cations [21, 22]. Most of these techniques have greatly reduced the required start-up period; however, the running cost is still expensive. Employing anaerobic granular sludge as seeding sludge can greatly reduce the required start-up time; however, the purchase and transportation of the granules are quite expensive [16].

The EGSB reactors in the present study were seeded with anaerobic flocculent sludge from the local POME treatment plant. Before the study, the system was operated in semicontinuous mode for 10 hr every day for one year [2]. Granulation did not appear even after an operation of one year.

During the current research, the cationic polymer (PAM) concentration fed to DAF unit was only about 15 mg/L in the first 17 weeks, while the average VFA concentration was 649.9 mg/L. Considering that half sludge was recycled to the dosing tanks, aerobic effluent average COD was 701.5 mg/L. From the 17th week on, PAM dose in DAF unit was increased to about 30 mg/L; consequently, the average VFA content reduced to 476 mg/L. Regulating the recycling of the half sludge to EGSB, the average effluent COD was 512 mg/L. After 23 weeks, the granulation of anaerobic sludge was evident. About 3 meters of anaerobic granular sludge developed in EGSB reactors after 23 weeks. Appropriate dose of cationic polymer (PAM) could accelerate the granulation of anaerobic sludge in spite of very high SS in the wastewater.

Basri et al. [23] reported the biomass wash out from the 500 m^3^ digester during anaerobic treatment of POME caused by the continuous recirculation of effluent. It was recommended that the mixing pump should be stopped at least 2-3 h prior to treating fresh POME so that sludge may be settled down and its wash out could be minimized. Appropriate mixing intensity is crucial during anaerobic treatment of POME.

A poor segregation of anaerobic granular sludge (better settleable), flocculent sludge (poor settleable), and SS may lead to sudden sludge flotation and reactor failure, especially at high organic loading rates (OLR). In addition, slower hydrolysis and the accumulation of inert substrate ingredients would induce a dilution of the active biomass to its lower specific activity during anaerobic digestion of SS-rich wastewaters. Pretreatment was recommended to eliminate a significant part of SS from the influent [24].

Latif et al. [25] reported that the COD removal efficiency declined at the SS loading rate was above 2.6 kg/m^3^/d, because relatively high SS levels probably disturbed the hydrolysis of the anaerobic digestion. Choi et al. [4] also recommended the pretreatment of POME in order to reduce SS concentration below 3000 mg/L to ensure better performance and stability of the anaerobic hybrid reactor (AHR).

An increasing accumulation of inorganic matter was noted in EGSB seeded with anaerobic granular sludge in the present study during 135 d operation resulting in change of VSS/SS rate from 75% to 56% [5]. Sufficient recycling or mechanical mixing, biogas recirculation, or even effluent recirculation was suggested to maintain the stability of anaerobic reactor while treating POME [26, 27]. But some investigators argued that rapid mixing would bring down pH during start-up and thus may harm methanogenic activity, resulting in the performance instability. Further investigation on the effects of mixing should be explored to decide on a suitable mixing mode for the best digester performance [28, 29].

In this study, the volume of produced biogas was 27.65 times that of influent flow rate (see Table 3), so the biogas alone was sufficient to act as the “mixer.” Additionally, an innovative influent distributor was installed at the bottom of EGSB reactor which was advancement over the single influent nozzle [26, 27].

The total alkalinity (as CaCO_3_) of EGSB effluent was in range of 5448 mg/L (as CaCO_3_), which could maintain the system pH above 6.8 without dosing extra caustic. The vertical flow regime from reactor bottom to top could ensure the success of metabolic syntrophic relationship between acidogens, acetogens, and methanogens. During hydrolysis and acidogenesis, the microbial communities hydrolyze heterogeneous complex organics to monomers such as glucose and amino acids, which are subsequently metabolized to acetate, propionate, butyrate, lactate, ethanol, and so forth. Hydrogen-producing acetogenic bacteria (HPAB) convert volatile fatty acids (VFA), for example, propionic and butyric acids, produced to H_2_, CO_2_, and acetic acid. Finally, the methanogens convert these intermediates to methane and carbon dioxide. A slight imbalance in these metabolic pathways may disturb the “relay position” of these microorganisms resulting in the instable syntrophic relationships. Volatile fatty acids (VFAs) accumulation may lead to lowering of pH and ultimately permanent process failure. Final effluent VFA of the current EGSB remained around 537 mg/L (as acetic acid) which was indicative of the process stability.

The organic SS fraction has a high potential for biogas production which makes the process economically more feasible. In addition, pretreatment would generate more surplus sludge requiring disposal at additional cost. The hydrolysis of SS is the rate-limiting step during anaerobic digestion of POME. Compared to other researches, the present anaerobic pilot-scale industrial plant did not remove SS from raw POME; rather prolonged HRT of 9.8 d was applied to deal it. Other strategies included retaining bulk of sludge in the reactor through the three-phrase separator of EGSB reactor, dosing PAM in DAF unit to improve SS removal efficiency. SS (inert substrate ingredients and anaerobic biomass) from DAF were also recirculated to anaerobic unit which increased their “hydraulic retention time” in the reactor. This would increase the biodegradability ratio of SS in POME to overcome their accumulation and consequently could increase the methane yield. Appropriate dose of cationic PAM accelerated the granulation of anaerobic sludge at high SS.

In order to improve the biological treatment efficiency, Chou et al. [30] applied batch thermoalkaline pretreatments to convert the complex biorefractory particulate organic materials to readily biodegradable low-molecular weight compounds. Their maximum COD solubilization (82.63%) occurred under the optimum conditions, that is, 32.5°C and 8.83 g/L of NaOH for 41.23 h reaction time. Chaiprapat and Laklam [31] investigated the preozonated POME which not only improved COD removal but also obtained a more stable performance without pH adjustment of anaerobic process. COD removal efficiency of 88.56% of the present study implied that recirculation of the SS prolonged “hydraulic retention time” of SS which improved total COD removal at the same HRT.

The scanning electron micrographs (SEM) of the granular sludge from these two EGSB reactors were presented in Figure 3. The granules had an average diameter of 1–3.5 mm. The ultrastructure of the granules revealed that the bacterial species of the granules were morphologically different from those at the surface. A stratified structure appeared in the bacterial cells present within the granules. It appeared that heterogeneous long rod-shaped and filamentous bacteria dominated the outer layer (Figures 3(b) and 3(c)), while the interior of granules comprised rod-shaped and little coccid bacteria (Figures 3(d), 3(e), and 3(f)). Three cavities were observed on the exterior of the granules as shown in Figure 3(c). Similar phenomena were also observed during POME treatment in an up-flow anaerobic sludge-fixed film bioreactor [10] and a pilot-scale EGSB [5].

The surplus sludge could be recovered as biofertilizer which showed better nutritional values compared to the raw POME. The pot trials showed that the application of organic fertilizers derived from the surplus sludge could enhance the soil fertility much better than the fertilizer derived from raw POME [2]. Biofertilizers have been regarded as an alternative to chemical fertilizers to increase crop production in sustainable farming [32].

## 4. Conclusions

The anaerobic EGSB reactors operated at HRT of 9.8 d reduced COD on the average from 71179 to an average effluent COD of 3587 mg/L achieving removal efficiency of 94.89% when half of sludge was recycled in DAF. The amount of produced biogas was 27.65 m^3^ biogas/m^3^ POME. The biogas had a rather stable composition of 65–70% CH_4_, 25–36% of CO_2_, and 800–1500 ppm of H_2_S. Dosing 30 mg/L cationic PAM in DAF unit and recycling half of sludge accelerated the anaerobic sludge granulation. Bacilli and coccid bacteria were the dominant microorganisms in the interior of granules.

## Figures and Tables

**Figure 1:** The schematic diagram and photographic presentation of the industrial-scale pilot EGSB reactors.

**Figure 2:** The variations on COD concentration and removal efficiency.

**Figure 3:** Scanning electron micrographs (SEM) of granular sludge from EGSB showing the predominant bacterial groups: (a) morphology of an overall anaerobic granules (65x magnification); (b) the exterior of anaerobic granules (5,000x magnification); (c) the cavities on the exterior of anaerobic granules (7,500x magnification); (d) the inner of anaerobic granules (7,500x magnification); (e) the inner structure of anaerobic granules (15,000x magnification); (f) the inner of anaerobic granules (10,000x magnification).

**Table 1:** Characteristic and composition of raw POME.

Parameter	Source a	Source b
Temperature (°C)	80–90	ND
pH	4.2	4.5 ± 1.19
Chemical oxygen demand (COD)	51000	76896 ± 119
Biochemical oxygen demand (BOD)	25000	27500 ± 100
Oil and grease (O & G)	6000	ND
Suspended solids (SS)	18000	27000 ± 82
Ammoniacal nitrogen (NH_3_-N)	35	36 ± 1
Total Kjeldahl nitrogen (TKN)	750	60 ± 6

Notes: Source a: [33]; Source b: [2].

All the measured parameters were expressed in mg/L, except pH and temperature. ND: not provided. Values present were the means of all determinations ± SD (standard deviation).

**Table 2:** The calculated data of POME samples.

Index (mg/L)	EQ tank	EGSB effluent	DAF effluent
BOD	30314 ± 1803	3564 ± 704	1335 ± 107
COD	71179 ± 8811	12341 ± 843	3587 ± 379
Suspended solids	32406 ± 2734	11456 ± 2734	1154 ± 82

Notes: all data are shown as means ± standard deviation of all samples.

**Table 3:** Evaluation of anaerobic EGSB for biogas production.

Parameter	Unit	Average value
2 EGSB total effective volume	m^3^	847.8
Capacity	m^3^/d	86.4 ± 4.1
Influent COD	mg/L	71179 ± 10950
EGSB effluent COD	mg/L	12341 ± 1338
DAF effluent COD	mg/L	3587 ± 546
EGSB effluent COD deduct recycled sludge	mg/L	7917 ± 955
Apparent COD removal efficiency	%	94.84 ± 1.08
Real COD removal efficiency	%	88.56 ± 1.97
Biogas production	m^3^/d	2389.0 ± 201.3
COD reduction	kg/d	5465.8 ± 259.4
Organic loading rate (OLR)	Kg COD/m^3^·d	6.45 ± 0.61
Efficiency (in POME injection)	m^3^ biogas/m^3^ POME	27.65 ± 3.02
Efficiency (in POME injection)	m^3^ biogas/kg COD	0.44 ± 0.04

Note: all data are shown as means ± standard deviation of all samples.
